The article "Sucrose-Formulated Recombinant Factor VIII Dosing Flexibility in Prophylaxis Regimens: Experience from Postmarketing Surveillance Studies" was published in 2015. Journal: Adv Hematol.

# Sucrose-Formulated Recombinant Factor VIII Dosing Flexibility in Prophylaxis Regimens: Experience from Postmarketing Surveillance Studies

**DOI:** 10.1155/2015/431268

**Published:** 2015-08-19

**Authors:** Thomas J. Humphries, Stephan Rauchensteiner, Claudia Tückmantel, Alexander Pieper, Monika Maas Enriquez, Prasad Mathew

**Affiliations:** ^1^Bayer HealthCare, 100 Bayer Boulevard, P.O. Box 915, Whippany, NJ 08981-0915, USA; ^2^Bayer Pharma AG, Global Medical Affairs Therapeutic Areas (GMA), Muellerstrasse 178, 13353 Berlin, Germany; ^3^Bayer Pharma AG, Aprather Weg 18a, Building 470, 42096 Wuppertal, Germany; ^4^M.A.R.C.O. GmbH & Co. KG, Moskauer Strasse 25, 40227 Düsseldorf, Germany; ^5^Bayer Pharma AG, Global Clinical Development Therapeutic Area NOHI, Aprather Weg, 42096 Wuppertal, Germany

## Abstract

*Objectives*. Prophylaxis regimens for severe hemophilia A allowing more flexible dosing while maintaining efficacy may improve adherence and decrease the cost of prophylaxis. Here, we compared the clinical effectiveness of once- or twice-weekly versus ≥3-times-weekly prophylaxis with sucrose-formulated recombinant factor VIII (rFVIII-FS) in a “real-world” practice setting. *Methods*. Data from 3 postmarketing studies were pooled. Patients with severe hemophilia A receiving ≥1 prophylaxis infusion/wk of rFVIII-FS for ≥80% of a prophylaxis observation period (≥5 months) were included. Patients were categorized based on physician-assigned treatment regimens of 1-2 prophylaxis injections/wk (*n* = 63) or ≥3 prophylaxis injections/wk (*n* = 76). Descriptive statistics were determined for annualized bleeding rates (ABRs). *Results*. Median (quartile 1; quartile 3) ABR for all bleeds was 2.0 (0; 4.0) in the 1-2 prophylaxis injections/wk group and 3.9 (1.5; 9.3) in the ≥3 prophylaxis injections/wk group. Median ABRs for joint, spontaneous, and trauma-related bleeds were numerically lower with 1-2 prophylaxis injections/wk. As an estimate of prophylaxis success, 63% (≥3 prophylaxis injections/wk) to 84% of patients (1-2 prophylaxis injections/wk) had ≤4 annualized joint bleeds. *Conclusions*. Dosing flexibility and successful prophylaxis with rFVIII-FS were demonstrated. Very good bleeding control was achieved with both once-twice-weekly and ≥3-times-weekly prophylaxis dosing regimens.

## 1. Introduction

Prophylaxis with factor VIII (FVIII) replacement products is the standard of care for patients with severe hemophilia in developed countries. Compared with on-demand treatment, prophylaxis confers several clinical benefits and is therefore recommended by World Federation of Hemophilia and National Hemophilia Foundation guidelines [1, 2]. However, standard prophylaxis generally requires injections ≥3 times per week [2], which can be a barrier to treatment adherence and may not be needed for all patients. Frequent infusions may be particularly challenging for young patients in whom venous access can be difficult [3]. Prophylaxis regimens that allow less frequent and more flexible dosing while maintaining efficacy may improve adherence and decrease the cost of prophylaxis.

The article "Sucrose-Formulated Recombinant Factor VIII Dosing Flexibility in Prophylaxis Regimens: Experience from Postmarketing Surveillance Studies" was published in 2015. Journal: Adv Hematol.

A number of studies have demonstrated the efficacy of sucrose-formulated recombinant FVIII (rFVIII-FS) using a ≥3-times-weekly dosing regimen [4–8]. Although only 2 prospective clinical studies have investigated the efficacy of rFVIII-FS using a once- or twice-weekly dosing regimen [9, 10], postmarketing studies of rFVIII-FS have collected data from patients using various prophylaxis regimens [11, 12]. Using pooled data from 3 postmarketing studies, the objective of this analysis was to compare the clinical effectiveness of once- or twice-weekly versus ≥3-times-weekly prophylaxis dosing with rFVIII-FS in patients with severe hemophilia A in the routine, or “real-world,” clinical setting.

## 2. Patients and Methods

Patients with hemophilia A included in this analysis receiving treatment with rFVIII-FS were enrolled in 1 of 3 postmarketing surveillance studies conducted in Austria, Denmark, France, Greece, Italy, Netherlands, Spain, Sweden [11], Taiwan [12], and Germany (KG0301-DE. Data on File, Berlin, Germany: Bayer Pharma AG, 2005). The studies included patients with hemophilia A who used rFVIII-FS for routine treatment for up to 24 months. For the current pooled analysis, patients with severe hemophilia with FVIII:C <1% who had a total prophylaxis observation period of ≥5 months and received ≥1 prophylaxis infusion per week for ≥80% of the prophylaxis observation period and who were considered valid for the efficacy analysis in the respective postmarketing surveillance study were selected. Patients with documented inhibitors or who were receiving rFVIII-FS for immune tolerance induction were excluded from the analysis. Data were collected in paper-based patient diaries during the postmarketing studies.

### 2.1. Dosing Regimens

The dosing regimen for each patient was determined by the treating physician. Patients who met the criteria for the pooled analysis were categorized into either the 1-2 prophylaxis injections/wk group, defined as 1 or 2 documented prophylaxis injections per week in ≥70% of the weeks during the prophylaxis observation period, or the ≥3 prophylaxis injections/wk group. In the real-world settings for these studies, presumably the treating physicians evaluated the global status of their patients before assigning dosing frequency.

The article "Sucrose-Formulated Recombinant Factor VIII Dosing Flexibility in Prophylaxis Regimens: Experience from Postmarketing Surveillance Studies" was published in 2015. Journal: Adv Hematol.

### 2.2. Data Collection and Analysis

Descriptive summary statistics were determined for demographic characteristics, the number of days in the prophylaxis observation period, number of prophylaxis injections per week, time between injections, prophylaxis dose per week, and the annualized bleeding rate (ABR) for total, joint, trauma-related, and spontaneous bleeding events. The results were analyzed overall and by the age subgroups of patients <18 versus ≥18 years.

Periods of prophylaxis treatment interruption (defined as no prophylaxis injection for >28 days) were excluded from the main analysis. Descriptive summary statistics were determined for the number of days excluded from the analysis based on this definition. In a sensitivity analysis, the number of exposure days and the ABR were analyzed for the total observation period from the first prophylaxis injection onward (i.e., including prophylaxis treatment interruptions) to assess the impact of excluded injections and bleeds that occurred during prophylaxis treatment interruption.

## 3. Results

### 3.1. Patients

Among 322 patients from the 3 postmarketing studies [11, 12] [KG0301-DE. Data on File, Berlin, Germany: Bayer Pharma AG; 2005], 139 were eligible for analysis based on the selection criteria for this analysis; 45% (*n* = 63) were grouped into the 1-2 prophylaxis injections/wk group and 55% (*n* = 76) were in the ≥3 prophylaxis injections/wk group. Of the 322 original patients, 183 (56%) were excluded from the pooled analysis for not fulfilling the criteria for prophylaxis treatment (*n* = 114), for having FVIII:C ≥1% (*n* = 57) or a history of inhibitors (*n* = 8), or for the fact that their rFVIII-FS use was for immune tolerance induction (*n* = 4). Demographic and prophylaxis dosing information by dosing group is shown in Table 1; overall, half of the patients were <18 years of age and most patients were white. The median (range) age was higher in the 1-2 prophylaxis injections/wk dosing group compared with the ≥3 prophylaxis injections/wk group (20 [0–63] years and 15 [1–71] years, resp.). Also, a higher percentage of patients aged <18 years were assigned to the ≥3 prophylaxis injections/wk group compared with the 1-2 prophylaxis injections/wk group (57% versus 44%). Fewer patients in the 1-2 prophylaxis injections/wk dosing group compared with the ≥3 prophylaxis injections/wk group had a target joint present at the time of enrollment into the respective studies (27% and 43%, resp., Table 1). This difference may be a result of physician evaluations prior to the assignment of dosing frequency.

### 3.2. Treatment

The median total prophylaxis observation time per patient was approximately 2 years (range, 140–839 days), and the majority of patients had no relevant prophylaxis treatment interruptions (nonprophylaxis periods, Table 1). The prophylaxis dose per week was lower in the 1-2 prophylaxis injections/wk group compared with the ≥3 prophylaxis injections/wk group. Patients in the 1-2 prophylaxis injections/wk group received an actual mean of 1.6 prophylaxis injections/week compared with 2.8 actual prophylaxis injections/wk for patients in the ≥3 prophylaxis injections/wk group. The mean annual dose for prophylaxis injections was 2300.1 IU/kg/y in the 1-2 prophylaxis injections/wk group and 3834.3 IU/kg/y in the ≥3 prophylaxis injections/wk group (Table 1).

The article "Sucrose-Formulated Recombinant Factor VIII Dosing Flexibility in Prophylaxis Regimens: Experience from Postmarketing Surveillance Studies" was published in 2015. Journal: Adv Hematol.

### 3.3. Prophylaxis Efficacy

The median (quartile 1; quartile 3 [Q1; Q3]) ABR for all bleeds was 2.0 (0; 4.0) in the 1-2 prophylaxis injections/wk group and 3.9 (1.5; 9.3) in the ≥3 prophylaxis injections/wk group (Figure 1); mean ± SD ABR was 4.1 ± 6.4 and 7.0 ± 10.7, respectively. Similarly, the median ABRs for joint bleeds, spontaneous bleeds, and trauma-related bleeds were numerically lower in the 1-2 prophylaxis injections/wk group compared with the ≥3 prophylaxis injections/wk group (Table 2).

When analyzed by age subgroup, the trend toward lower ABRs for all bleeds in the 1-2 prophylaxis injections/wk group was observed for both the <18 and ≥18 year subgroups (Table 3). However, the ABRs were higher in patients ≥18 years compared with patients <18 years. The lowest median ABR (Q1; Q3) for all bleeds was observed in patients <18 years receiving 1-2 prophylaxis injections/wk (1.9 [0; 3.0]), and the highest was observed in patients ≥18 years receiving ≥3 prophylaxis injections/wk (4.7 [1.9; 11.2]). The ABRs for joint and spontaneous bleeds were also higher in patients ≥18 years compared with patients <18 years in each dosing group, whereas the ABR for trauma-related bleeds was lower in patients ≥18 years compared with patients <18 years (Table 3).

A greater percentage of patients in the 1-2 prophylaxis injections/wk group had 0 annualized bleeds and 0 annualized joint bleeds compared with patients in the ≥3 prophylaxis injections/wk group (30% and 40% versus 7% and 17%, resp., Table 4). In the 1-2 prophylaxis injections/wk group, 81% had ≤8 annualized bleeds compared with 68% of patients in the ≥3 prophylaxis injections/wk group. For joint bleeds, 84% of patients in the 1-2 prophylaxis injections/wk group had ≤4 annualized joint bleeds compared with 63% of patients in the ≥3 prophylaxis injections/wk group. Patients in the 1-2 prophylaxis injections/wk group were still more likely to have 0 annualized bleeds, regardless of age subgroup (data not shown). However, the lower percentage of patients in the total population receiving 1-2 prophylaxis injections/wk with >8 annualized bleeds compared with patients in the ≥3 prophylaxis injections/wk group was only observed in patients <18 years. For joint bleeds, the frequency pattern was generally similar to the overall population, but there were more patients <18 years of age with 0 annualized joint bleeds compared with patients ≥18 years of age in both dosing groups.

The article "Sucrose-Formulated Recombinant Factor VIII Dosing Flexibility in Prophylaxis Regimens: Experience from Postmarketing Surveillance Studies" was published in 2015. Journal: Adv Hematol.

Analyses using different prophylaxis regimen definitions (receiving 1-2 or ≥3 prophylaxis injections/wk in 50% of the weeks during the observation period versus 70%) resulted in similar results as the primary analysis. A sensitivity analysis included the total observation time from the first prophylaxis injection until the end of the observation time irrespective of any interruption of prophylaxis treatment. The reason for this sensitivity analysis was to make sure that bleeding treatment periods were not wrongly interpreted as interruptions of prophylaxis treatment. Results from this analysis showed that there were no major changes in bleeding results and, especially, that the approach of the primary analysis did not introduce bias in favor of the 1-2 prophylaxis injections/wk group.

## 4. Discussion

In this pooled analysis of data from 3 postmarketing studies, 1-2 weekly infusions of rFVIII-FS were at least as effective as ≥3-times-weekly dosing in preventing bleeding episodes in patients with severe hemophilia A, demonstrating effective prophylaxis dosing flexibility with rFVIII-FS for some patients under real-life conditions. Almost half of the patients (45%) treated with prophylaxis were using a regimen of 1-2 prophylaxis injections/wk; adult patients and patients without target joints were more likely to be prescribed this regimen. The median ABR for all, joint, trauma-related, and spontaneous bleeds was numerically lower for patients receiving 1-2 prophylaxis injections/wk compared with those receiving ≥3 prophylaxis injections/wk. Furthermore, the percentage of patients with 0 bleeding episodes was higher in the 1-2 prophylaxis injections/wk group compared with the ≥3 prophylaxis injections/wk group.

In these postmarketing studies, dosing frequency was assigned by the treating physician. Patients following a 1-2 prophylaxis injections/wk regimen may have had a milder bleeding phenotype, had fewer target joints, or had other factors that influenced FVIII half-life; therefore, patients in this group may have been less prone to bleeds in general or experienced a longer duration of protection from bleeding, resulting in numerically better outcomes compared with patients treated ≥3 times/wk. Bleeding history information, such as the number of bleeding episodes in the previous year, was not available to investigate this hypothesis. However, since physicians base their treatment assignment in clinical practice on specifics of patient medical history and characteristics, it can be assumed that the assignment to a lower frequency of prophylaxis occurred for those patients with a milder bleeding phenotype in the past. The effect of different types of prophylaxis regimens on joint outcomes was not the subject of this analysis. The fact that the percentage of patients with target joints was lower in the 1-2 prophylaxis injections/wk group compared with the ≥3 prophylaxis injections/wk group suggests that the lower frequency regimen was most likely assigned to patients with a milder bleeding phenotype. Indeed, results from a randomized, double-blind study indicated that, while receiving 3-times-weekly prophylaxis with rFVIII-FS, significantly more bleeds were reported in patients with target joints versus without target joints [4].

The article "Sucrose-Formulated Recombinant Factor VIII Dosing Flexibility in Prophylaxis Regimens: Experience from Postmarketing Surveillance Studies" was published in 2015. Journal: Adv Hematol.

Analysis by age subgroup revealed that the trend toward lower ABRs observed in the 1-2 prophylaxis injections/wk group compared with the ≥3 prophylaxis injections/wk group was not age dependent. However, there was a trend toward higher joint bleeding rates in patients ≥18 years of age compared with patients <18 years of age and more trauma-related bleeds in the lower age group. An analysis of bleeding patterns in patients with severe hemophilia A receiving prophylaxis during prospective clinical trials found lower bleeding rates in adults compared with children [13]. However, this same analysis also reported a trend toward increasing frequency of joint bleeds with increasing age and higher trauma-related bleeding rates in children [13], which is in agreement with the results of this pooled analysis.

The data from this pooled analysis support the hypothesis that not all patients need the standard 3-times-weekly dosing regimen to achieve bleeding control [14]. This hypothesis is further supported by data from the Canadian Hemophilia Primary Prophylaxis (CHPS) study, a prospective, long-term study that investigated the efficacy of tailored prophylaxis for severe hemophilia A [10]. Of the 56 boys in the study at study year 13, 36 (64%) had escalated from once-weekly prophylaxis to twice-weekly prophylaxis to control bleeding; 17 of these 36 patients escalated from twice-weekly prophylaxis to alternate-day prophylaxis [15, 16].

A limitation of this analysis is that the data are pooled from observational, noninvestigational “real-world” studies. The results must be considered without pharmacokinetic data or data on time to fall below a certain FVIII trough level. In addition, historical bleeding data are not available to investigate possible reasons for the differences in bleeding rates observed between the 2 dosing groups nor is information available on the treating physicians' rationale for selecting a specific dosing frequency. Also, unlike the CHPS study, joint outcomes were not assessed in the current study, and only annualized bleeding rates were evaluated. Another potential limitation of the analysis was that periods without documentation of injections or bleeds could have biased results or assignment of patients to analysis groups. To avoid this bias, periods of prophylaxis treatment interruption ≥28 days were excluded from the analysis. A cut-off threshold of 28 days is theoretically a long enough time period to be representative of a true prophylaxis treatment interruption without excluding data from bleeding treatment periods; however, it was possible that some bleeds may have required treatment for >28 days. A sensitivity analysis that included all data during the prophylaxis treatment interruptions showed no major differences compared with the primary analysis.

The article "Sucrose-Formulated Recombinant Factor VIII Dosing Flexibility in Prophylaxis Regimens: Experience from Postmarketing Surveillance Studies" was published in 2015. Journal: Adv Hematol.

A definition of successful prophylaxis in the clinical practice setting has not yet been determined. In these postmarketing data, 81% of the once-twice-weekly dosing group had ≤8 total annualized bleeds compared with 68% of those in the ≥3-times-weekly dosing group. The results for annualized joint bleeds, perhaps a better gauge of prophylaxis success, were 84% and 63% for ≤4 joint bleeds for the 2 groups, respectively. In the absence of data on patient adherence, these results might be considered successful prophylaxis in a practice setting. Nevertheless, one-third of the patients treated with a standard prophylaxis regimen of 3x/week did not demonstrate an acceptable outcome of joint bleed control with the dosages used for prophylaxis injection. A possible explanation is the difference in incidence of target joints at baseline between the dosing groups. In patients <12 years of age, target joints at baseline were present in 5.9% in the once-twice-weekly group versus 22.6% in the ≥3-times-weekly group. The corresponding figures for those ≥12 years of age were 34.8% versus 57.8%. It can only be speculated that higher dosages may provide better outcomes in terms of prevention of joint bleeds in these patients.

## 5. Conclusions

Dosing flexibility with rFVIII-FS was demonstrated in this pooled analysis from 3 postmarketing studies. Very good bleeding control as shown by ABR for all bleeds and joint bleeds was achieved by both a standard ≥3-times-weekly dosing regimen and by a less frequent once-twice-weekly regimen. The prophylaxis success achieved was reasonable in the absence of an agreed definition of success in the clinical setting. The selection of dosing regimen was made by the treating physician. The patients prescribed the less frequent regimen were likely to be older and to be without target joints.

The article "Sucrose-Formulated Recombinant Factor VIII Dosing Flexibility in Prophylaxis Regimens: Experience from Postmarketing Surveillance Studies" was published in 2015. Journal: Adv Hematol.

## Figures and Tables

**Figure 1:** Annualized bleeding rate for all bleeds by dosing group. Q1 = quartile 1; Q3 = quartile 3.

**Table 1:** Demographic and dosing characteristics.

	Prophylaxis 1-2x/wk (*n* = 63)	Prophylaxis ≥3x/wk (*n* = 76)	Total (*N* = 139)
Age, y			
Mean	23	21	22
Median (range)	20 (0–63)	15 (1–71)	17 (0–71)
<18 y, *n* (%)	28 (44)	43 (57)	71 (51)
Race, *n* (%)			
White	52 (83)	61 (80)	113 (81)
Asian	5 (8)	4 (5)	9 (7)
Others	2 (3)	3 (4)	5 (4)
Missing	4 (6)	8 (11)	12 (9)
Target joint present, *n* (%)	17 (27)	33 (43)	50 (36)
Prophylaxis observation period, d			
Mean ± SD	573 ± 220	609 ± 207	593 ± 213
Median (range)	695 (151–826)	731 (140–839)	726 (140–839)
Number of excluded nonprophylaxis days/patient^*∗*^			
Mean ± SD	41 ± 108	34 ± 96	37 ± 101
Median (range)	0 (0–516)	0 (0–506)	0 (0–516)
Number of all injections/wk/patient			
Mean ± SD	1.8 ± 0.5	3.1 ± 0.5	2.5 ± 0.8
Median (range)	1.9 (1.0–3.2)	3.0 (2.0–4.8)	2.6 (1.0–4.8)
Number of prophylaxis injections/wk/patient			
Mean ± SD	1.6 ± 0.4	2.8 ± 0.4	2.3 ± 0.7
Median (range)	1.6 (0.9–2.2)	2.8 (1.5–3.8)	2.3 (0.9–3.8)
Time between prophylaxis injections,^†^ d			
Mean ± SD	4.4 ± 1.4	2.2 ± 0.4	3.2 ± 1.5
Median (range)	4.0 (3.0–7.0)	2.0 (2.0–3.0)	3.0 (2.0–7.0)
Prophylaxis dose/wk, IU/kg			
Mean ± SD	44.1 ± 26.8	73.5 ± 33.9	60.2 ± 34.1
Median (range)	33.5 (11.4–101.9)	71.5 (17.1–166.5)	56.2 (11.4–166.5)
Prophylaxis dose/injection, IU/kg			
Mean ± SD	27.0 ± 13.5	26.2 ± 11.2	26.6 ± 12.2
Median (range)	26.6 (6.3–56.4)	27.0 (6.5–54.2)	26.9 (6.3–56.4)
Prophylaxis dose/y, IU/kg			
Mean ± SD	2300.1 ± 1396.5	3834.3 ± 1768.9	3139.0 ± 1778.8
Median (range)	1750.3 (594.8–5318.1)	3732.8 (890.7–8687.3)	2930.6 (594.8–8687.3)

^*∗*^Interruptions in prophylaxis treatment, defined as periods of ≥28 days without any prophylaxis injection, were excluded from the main analysis.

^†^Median time per patient between 2 prophylaxis infusions was analyzed.

**Table 2:** Annualized bleeding rates by dosing group.

Annualized bleeding rates	Prophylaxis 1-2x/wk (*n* = 63)	Prophylaxis ≥3x/wk (*n* = 76)
All bleeds		
Mean ± SD	4.1 ± 6.4	7.0 ± 10.7
Median (Q1; Q3)	2.0 (0; 4.0)	3.9 (1.5; 9.3)
Joint bleeds		
Mean ± SD	2.8 ± 5.2	4.5 ± 7.0
Median (Q1; Q3)	0.9 (0; 2.6)	2.4 (0.6; 5.5)
Spontaneous bleeds		
Mean ± SD	2.4 ± 5.0	3.1 ± 6.2
Median (Q1; Q3)	0 (0; 1.9)	0.9 (0; 3.7)
Trauma-related bleeds		
Mean ± SD	1.6 ± 3.7	3.4 ± 5.4
Median (Q1; Q3)	0.6 (0; 2.0)	1.5 (0.5; 4.6)

Q1 = quartile 1; Q3 = quartile 3.

The article "Sucrose-Formulated Recombinant Factor VIII Dosing Flexibility in Prophylaxis Regimens: Experience from Postmarketing Surveillance Studies" was published in 2015. Journal: Adv Hematol.

**Table 3:** Annualized bleeding rates by dosing and age subgroups.

Annualized bleeding rates	Prophylaxis		Prophylaxis	
	1-2x/wk		≥3x/wk	
	(*n* = 63)		(*n* = 76)	
	Age <18 y *n* = 28	Age ≥18 y *n* = 35	Age <18 y *n* = 43	Age ≥18 y *n* = 33
All bleeds				
Mean ± SD	3.0 ± 5.6	5.0 ± 6.9	5.8 ± 5.9	8.7 ± 14.7
Median (Q1; Q3)	1.9 (0; 3.0)	2.4 (0; 8.4)	3.5 (1.1; 8.5)	4.7 (1.9; 11.2)
Joint bleeds				
Mean ± SD	1.5 ± 3.4	3.9 ± 6.1	2.9 ± 3.2	6.6 ± 9.6
Median (Q1; Q3)	0.5 (0; 1.5)	1.7 (0; 3.5)	1.8 (0.5; 4.2)	3.8 (1.5; 8.5)
Spontaneous bleeds				
Mean ± SD	0.5 ± 1.0	3.9 ± 6.3	1.1 ± 2.2	5.8 ± 8.5
Median (Q1; Q3)	0 (0; 0.5)	1.1 (0; 6.8)	0.5 (0; 1.0)	3.0 (0; 8.8)
Trauma-related bleeds				
Mean ± SD	2.4 ± 5.1	1.1 ± 1.9	4.3 ± 4.5	2.4 ± 6.2
Median (Q1; Q3)	1.0 (0; 2.4)	0 (0; 1.1)	2.5 (0.9; 7.0)	0.7 (0; 1.9)

Q1 = quartile 1; Q3 = quartile 3.

**Table 4:** Annualized bleeding frequency.

	Number (%) of patients		
	Prophylaxis 1-2x/wk (*n* = 63)	Prophylaxis ≥3x/wk (*n* = 76)	Total (*N* = 139)
Total bleeds			
0	19 (30.2)	5 (6.6)	24 (17.3)
>0 to ≤2	12 (19.0)	19 (25.0)	31 (22.3)
>2 to ≤8	20 (31.7)	28 (36.8)	48 (34.5)
>8	12 (19.0)	24 (31.6)	36 (25.9)
Joint bleeds			
0	25 (39.7)	13 (17.1)	38 (27.3)
>0 to ≤2	18 (28.6)	23 (30.3)	41 (29.5)
>2 to ≤4	10 (15.9)	12 (15.8)	22 (15.8)
>4	10 (15.9)	28 (36.8)	38 (27.3)
